# Testing an individualized digital decision assist system for the diagnosis and management of mental and behavior disorders in children and adolescents

**DOI:** 10.1186/s12911-020-01239-2

**Published:** 2020-09-17

**Authors:** Carolyn E. Clausen, Bennett L. Leventhal, Øystein Nytrø, Roman Koposov, Odd Sverre Westbye, Thomas Brox Røst, Victoria Bakken, Kaban Koochakpour, Ketil Thorvik, Norbert Skokauskas

**Affiliations:** 1 Regional Center for Child and Youth Mental Health and Child Welfare (RKBU)- Central Norway, IPH, Faculty of Medicine and Health Sciences, The Norwegian University of Science and Technology (NTNU), Trondheim, Norway; 2 Division of Child and Adolescent Psychiatry, Department of Psychiatry, The University of California San Francisco (UCSF), San Francisco, California USA; 3 Department of Computer Science, Faculty of Information Technology and Electrical Engineering, The Norwegian University of Science and Technology (NTNU), Trondheim, Norway; 4 Regional Center for Child and Youth Mental Health and Child Welfare (RKBU)- Northern Norway, UiT The Arctic University of Norway, Tromsø, Norway; 5 Sechenov First Moscow State Medical University, Moscow, Russia; 6 Department of Child and Adolescent Psychiatry, St. Olavs Hospital, Trondheim, Norway; 7 Central Norway Regional Health Information Technology (HEMIT), Trondheim, Norway

**Keywords:** Child and adolescent mental health services (CAMHS), Clinical decision support system (CDSS), Innovation, Attention-deficit/hyperactivity disorder (ADHD), IDDEAS, Norway

## Abstract

**Background:**

Nearly half of all mental health disorders develop prior to the age of 15. Early assessments, diagnosis, and treatment are critical to shortening single episodes of care, reducing possible comorbidity and long-term disability. In Norway, approximately 20% of all children and adolescents are experiencing mental health problems. To address this, health officials in Norway have called for the integration of innovative approaches. A clinical decision support system (CDSS) is an innovative, computer-based program that provides health professionals with clinical decision support as they care for patients. CDSS use standardized clinical guidelines and big data to provide guidance and recommendations to clinicians in real-time. IDDEAS (Individualised Digital DEcision Assist System) is a CDSS for diagnosis and treatment of child and adolescent mental health disorders. The aim of IDDEAS is to enhance quality, competency, and efficiency in child and adolescent mental health services (CAMHS).

**Methods/design:**

IDDEAS is a mixed-methods innovation and research project, which consists of four stages: 1) Assessment of Needs and Preparation of IDDEAS; 2) The Development of IDDEAS CDSS Model; 3) The Evaluation of the IDDEAS CDSS; and, 4) Implementation & Dissemination. Both qualitative and quantitative methods will be used for the evaluation of IDDEAS CDSS model. Child and adolescent psychologists and psychiatrists (*n* = 30) will evaluate the IDDEAS` usability, acceptability and relevance for diagnosis and treatment of attention-deficit/hyperactivity disorder.

**Discussion:**

The IDDEAS CDSS model is the first guidelines and data-driven CDSS to improve efficiency of diagnosis and treatment of child and adolescent mental health disorders in Norway. Ultimately, IDDEAS will help to improve patient health outcomes and prevent long-term adverse outcomes by providing each patient with evidence-based, customized clinical care.

**Trial registration:**

ISRCTN, ISRCTN12094788. Ongoing study, registered prospectively 8 April 2020 10.1186/ISRCTN12094788

## Background

Mental health disorders today account for more years lived with disability (YLDs) than any other health condition, with close to 30% of all people worldwide having a mental health disorder at one point during their lifetimes [1, 2]. Children and adolescents are particularly vulnerable. Nearly 20% of all children and adolescents at any point in time have a diagnosable mental health disorder [3, 4]. Despite this, no more than one-third of all children and adolescents with mental health disorders worldwide receive the care they require [5].

In Norway, approximately 20% of all children and adolescents are experiencing mental health problems at any point in time [6, 7]. Both, academic pressure at school and social pressure among peers, contribute to children and adolescents reporting more stress now than ever before [8]. While primary care providers (PCPs) often serve as the first point of contact for patients and their families, still most PCPs do not hold adequate training to address complex neuropsychiatric disorders, such as autism spectrum disorder (ASD) and attention-deficit/hyperactivity disorder (ADHD) [9–12].

Inability to receive a timely diagnosis and appropriate early intervention for neuropsychiatric disorders in childhood and adolescence leads to higher risk of suffering from comorbid mental health problems, including alcohol and substance abuse, behavioral problems [9, 13]. Insufficient access to required child and adolescent mental health services (CAMHS), not only directly impacts the health of the patients and their families, but also can be costly for the society as a whole [14–16]. Misdiagnosed or untreated mental health problems in childhood and adolescence can develop into lifelong mental health disorders requiring long-term care services. Across the European Union, the annual accumulated cost of providing mental health care for children and adolescents is estimated to be nearly €21 billion [16]. Undiagnosed or untreated disorders are also detrimental to the society’s future job market and economic stability, with more frequent work absences and lower productivity among individuals struggling with long-term mental illness [17].

Every year, roughly 5% of the child and adolescent population in Norway require specialist care from CAMHS [18, 19]. Among Norwegian twelve-year-olds alone, an estimated 3.4% have ADHD at any point in time; it is one of the most common reasons for referral to CAMHS [18]. If left untreated, ADHD can predispose children and adolescents to psychiatric and social pathology later in life [20, 21]. While Norway ensures every citizen to timely care by law [22], it is essential to optimize the quality of diagnostics and early intervention care for all children and adolescents displaying signs of mental illness. One modern approach to CAMHS quality assurance, that has the potential to be cost efficient and sustainable for long-term needs, is the incorporation of information and communication technologies (ICT), including clinical decision support systems (CDSSs) [23, 24].

A CDSS is a computerized system that offers guidance to clinicians in real-time while they provide clinical care by using existing, evidence based resources [25–27]. A CDSS uses compiled evidence-based resources to provide clinicians with clinically relevant guidance and recommendations to help best meet the needs of each individual patient. CDSSs are not designed to replace clinicians. The architecture of a CDSS typically has three distinct components– a Clinical Knowledge Base (domain of expertise based on clinical guidelines and/or health datasets), a Reasoning Engine (cloud based organization of evidence relative to the patient’s electronic health record (EHR)), and a User-Interface (electronic display that provides alerts and recommendations in response to clinician’s queries) [13, 27]. CDSS model designs however can differ; utilizing standardized clinical guidelines (i.e., DSM-V or ICD-11), and/or aggregated health datasets [27]. A CDSS that uses guidelines translates the guidelines into web ontology language (OWL) modeled computerized-guidelines as the base for clinical guidance. CDSSs that incorporate health datasets, also known as “data-driven” CDSSs, use algorithms and data analytics to identify patterns of care trajectories that are relevant to the patient being seen [28–30]. While both approaches have relative strengths, a CDSS model that is both guideline based and data-driven also allows the clinician to receive evidence-based support that is customized to each individual patient, based on extensive evidence and previous patient cases [27–30].

While CDSS implementation in general medicine has been found to be advantageous for the quality of services [30, 31], there is limited evidence on the use of CDSSs for CAMHS [32]. One reason for such limited research is the lack of accessibility to psychiatric data, especially those pertaining to children and adolescents. From the established studies on CDSSs in CAMHS however, most have identified various limitations, including a lack of integration with the EHR, limited predictive models for diagnosis, and inadequate inclusion of multiple disorders [32]. Norway is in a unique position to develop and implement a CDSS for CAMHS because it can potentially avoid previously identified limitations. Over the past decade, the Norwegian National Association of Child and Adolescent Mental Health (N-BUP), has collected extensive data on CAMHS and compiled unique and rich datasets, based on advanced, multidisciplinary EHRs. However, these datasets have yet to be optimally utilized for subsequent care, as maintaining access requires ethical clearance and completion of a local data protection impact assessment (DPIA) and risk assessment to ensure privacy and confidentiality will not be breached.

This paper presents the study design and protocol for the evaluation of the first CDSS for CAMHS in Norway, the Individualized Digital Decision Assist System (IDDEAS). IDDEAS is an innovative research project, contributing to the HELSEVEL Programme (Programme on Health, Care and Welfare Services Research) and funded by the Norwegian Research Council (NFR). The overall aim of IDDEAS is to improve patient care by providing practitioners with real-time, data-driven and evidence-based guidance that ensures earlier and more precise decision-making, avoids misdiagnosis and reduces inefficiency in patient care practices. The principal benefit of the study is to examine the provision of decision support for clinicians in real-time during clinical sessions and improvement of clinical care.

The objectives of the IDDEAS project include:

1. Evaluate the clinical utility of IDDEAS for diagnosis and treatment of child and adolescent mental health disorders
2. Measure clinicians’ perceived clinical usability and appropriateness of IDDEAS for child and adolescent mental health care
3. Measure the clinical relevance and validity of IDDEAS’ user-interface content for clinical care
4. Implement IDDEAS in local Norwegian CAMHS and establish recommendations for future CDSS design and implementation for child and adolescent mental health disorders

## Methods

### Study design and process

The IDDEAS project is an experimental, mixed-methods evaluation study, within CAMHS in Norway. The study evaluates the IDDEAS CDSS model (see Fig. 1) for diagnosis and treatment in CAMHS in Norway; IDDEAS will use ADHD as the first clinical model paradigm. The study consists of the following four stages:

**Fig. 1:** The IDDEAS Clinical Decision Support System Model

*Stage 1: The Assessment of Needs & Preparation of IDDEAS.*

*Stage 2: The Development of the IDDEAS CDSS Model.*

*Stage 3: The Evaluation of the IDDEAS CDSS.*

*Stage 4: Implementation & Dissemination.*

### Stage 1: assessment of needs and preparation of IDDEAS

The preparation of IDDEAS includes the establishment of the IDDEAS Consortium, completion of a stakeholder analysis, clinical guidelines and clinical case vignettes validation, and the user-interface design and modeling. The IDDEAS Consortium consists of local CAMHS clinicians, international CAMHS experts, CDSS and software experts, as well as representatives from various service-user organizations (i.e., ADHD Norge, Bikuben, The National Association for Relatives in Mental Health- LPP Tromsø, etc.).

#### IDDEAS stakeholder validation of clinical guidelines and case vignettes

IDDEAS Consortium will first hold a discussion of the current status of CAMHS in Norway and validate the standardized clinical practice guidelines for inclusion within the IDDEAS CDSS, as well as the clinical case vignettes to be used to evaluate the IDDEAS CDSS model. The IDDEAS Consortium will employ clinicians and CAMHS experts as external collaborators for the validation processes. The fictional clinical case vignettes will be created by the IDDEAS Consortium and will be considered valid fictional representations of patient cases with majority consensus (*n* = 10). Both, the guidelines and the clinical case vignettes will be discussed and validated in collaborative focus group discussions held at the Regional Center for Child and Youth Mental Health and Child Welfare (RKBU), Central Norway in Trondheim, Norway. The clinicians in attendance will not participate in the evaluation of IDDEAS to avoid exposure bias and will receive compensation for their time.

#### IDDEAS user-Interface design

As the final part of the IDDEAS preparation, the IDDEAS IT team will collaborate with the Consortium’s clinicians (i.e., local and international CAMHS experts) to design the IDDEAS CDSS user-interface. The IDDEAS IT team will conduct focus groups with the CAMHS experts in order to identify what is most important to address with the design of the user-interface to ensure sufficient usability and acceptability. The IDDEAS CDSS user-interface will be integrated within the patient’s EHR to display prompts and alerts for clinicians in real time.

### Stage 2: development of the IDDEAS CDSS model

Following the validation of the clinical guidelines and clinical case vignettes, and the development of the IDDEAS user-interface design in Part 1, the model of the system will be developed. The previously collected health datasets (i.e., *BUP-data*) to be included in the Clinical Knowledge Base will be aggregated and de-identified. The IDDEAS research team will follow all formal data protection procedures, including the completion of the local DPIA and risk assessment (i.e. ROS Analysis). The datasets will be de-identified using a list of personal identifiers (PID) data placeholders established by the local IDDEAS research team. Prior to integration of the de-identified data within the model, the IDDEAS IT team will internally test the reliability and functionality of the PID placeholders for adequate de-identification of the health datasets.

As the last step in the IDDEAS CDSS development process, prior to the evaluation of the IDDEAS CDSS model, the functionality of the Reasoning Engine will be tested. The IDDEAS Consortium will collaboratively create a list of clinical competence questions (CCQs) based on a previously validated fictional patient case. The CCQs will be input into the user-interface to simulate a clinician querying the system during a clinical session. The utility of the Reasoning Engine will be assessed based on whether the system optimally receives the CCQs, and returns a set of evidence-based, ranked, recommendations for diagnosis and treatment.

### Stage 3: evaluation of the IDDEAS CDSS model

#### Recruitment and eligibility

Study participants are child and adolescent psychiatrists and psychologists (*n* = 30). Participants will represent four child and adolescent mental health clinics (BUP-clinics); the clinics will be chosen at random in collaboration with the N-BUP (Norwegian Association for Child and Adolescent Psychiatry) representative. Purposive sampling will be undertaken to ensure there is a balance among participants, in regards to gender, location in the country, expertise and socioeconomic status. This approach to sampling will limit bias and ensure inclusion of varied perspectives. Recruitment of participants for enrollment in the study will begin no earlier than August 2020. Participants are deemed eligible if they are currently practicing as a child and adolescent psychologist or psychiatrist in Norway.

#### Sample size

The sample size was calculated based on the optimal power value in order to ensure the size of the sample is appropriate for this study. There is the assumption that the effect of decision support is to increase specificity from 0.50 to 0.80 and only moderately change sensitivity. With the assumption that the effect of decision support is to increase specificity from 0.50 to 0.80 and only moderately change sensitivity, the sample size (*n* = 30) can be calculated with an effect size of at least 1.0 and desired power value of .80 (80%); the assumption of the specificity increase, to detect the statistical significance (*p* < 0.05) on a dichotomous variable with 80% power, the number of subjects required is 30.

#### Procedure

The evaluation of the CDSS model initially will entail assessments of how child and adolescent psychologists and psychiatrists perceive the usability, acceptability, validity, and relevance of the CDSS model for use in their clinical practice. The evaluation of the CDSS model will take place in two phases, as follows: Phase 1. Vignette-Based Evaluation and Phase 2. Live Patient Evaluation. Both phases of the CDSS evaluation will occur in randomly selected CAMHS clinics. The incremental evaluation phases will take place within the trial period of August 2020–2023. Using a pre-post design, for both phases of the evaluation, participants will compare the provision of clinical care with use of the CDSS, to the daily clinical practice, as the control. Prior to participation in the evaluation written consent will be obtained from all participants by the project leader. Participants will be informed their participation is voluntary and they can withdraw from the study at any time without penalty.

##### Phase 1: vignette-based evaluation

After completion of informed consent procedures, including assessments of conflicts of interest, clinicians will be asked to complete a brief demographic questionnaire. They will then be provided the educational manual on how to navigate the IDDEAS system. Clinicians will then be asked to critically appraise ten previously validated clinical case vignettes (i.e., fictional patient cases that have been “referred” for assessment of ADHD). Clinicians will first appraise five of the cases without the use of the system and five using the CDSS. The cases will be randomly allocated by the PhD student with the project and verified by the project leader. The allocation sequence will be computer generated.

##### Phase 2: live patient evaluation

Phase 2 will entail a live patient evaluation study of the IDDEAS CDSS model for the diagnosis and treatment of ADHD among children and adolescents in which seven standardized patient-encounter videos will be assessed with and without the use of the IDDEAS system. The aim of this phase of the study is to determine whether IDDEAS in its entirety can: meet the desired requirements; can yield an output that meets specifications with acceptable capability.

#### Data collection

##### Qualitative methods

All participants will be surveyed using both qualitative and quantitative methods. In the vignette-based evaluation, all participants will be asked to complete a “cognitive- walkthrough” in which they will think-aloud through the entire process of critically appraising each clinical vignette case. In the live patient evaluation, the same procedure will be conducted to evaluate clinical care with the CDSS, based on seven standard patient encounter videos. All participants will be queried with a semi-structured interview in order to gain understanding of the participants’ overall experience, challenges encountered, strengths, and any other aspects of the system requiring adjustment. The semi-structure interviews will be held directly after the completion of the case vignettes. For both phases of the evaluation, the cognitive-walkthrough and semi-structured interview will be audio recorded and transcribed. Transcripts will be transferred to NViVo 10 software for coding and data analysis [33, 34].

##### Quantitative methods

All quantitative measurements will be translated from English to Norwegian as needed and compiled into an assessment package in accordance with the WHO’s guideline “Process of Translation and Adaptation of Instruments” (see Table 1) [35]. Data will also be collected on the sensitivity, specificity, and relevance of the IDDEAS system. Data will be collected on standardized score sheets, transferred to a Microsoft Excel spreadsheet, and retained/stored in a database system serving as a scalable informatics framework (i.e., Informatics for Integrating Biology & the Bedside (i2b2)) for subsequent analysis. The database system will provide an ontology-based flexibility that enables aggregation of multiple datasets, as well as easy extraction of individual clinical cases. All participants’ demographic information will also be anonymized with a randomly assigned unique study ID, aggregated and encrypted prior to transfer to a secure data repository for storage. Access to participants’ demographic information and study IDs will only be available to the IDDEAS project leader and the PhD student affiliated with the project. Datasets will be stored in a secure data repository at the Regional Center for Child and Youth Mental Health and Child Welfare (RKBU), Department of Mental Health, Norwegian University of Science and Technology (NTNU).

**Table 1:** Quantitative Assessment Measurements

Full Name	Abbreviation	About	Measure
System Usability Scale	SUS	To establish each participant’s individual rating score of usability aspects (e.g. the ability of users to complete tasks, level of resources/effort needs for task completion, and user’s subjective reaction to the system.)	Perceived Usability
User-Engagement Scale	UES	Measure user engagement with the system, including: appropriateness for clinical session, focused attention, aesthetics appeal, and felt involvement	Appropriateness
Content Validity Index	CVI	To capture inter-rater agreement on the relevance and appropriateness of each proposed item.	Relevance

#### Data analysis

##### Qualitative methods

For both phases of the evaluation, the semi-structured interviews and the “cognitive- walkthrough” recordings, will both be analyzed using thematic (i.e., Grounded Theory) and content analysis. The thematic analysis will identify patterns within the participants’ transcribed response to identify attributes of the overall appropriateness, including: challenges experienced assessing the cases, limitations in the interactive component of the system, strengths of the system’s design, and potential additions to the system’s design in order to improve the experience. Content analysis will be used to assess the frequency of items and prompts used during the interviews [33, 36, 37].

##### Quantitative methods

The Likert scale items will be assessed based on inter-rater reliability in accordance with pre-specified and previously validated criteria. The usability, content validity, and user engagement data will be compiled and analyzed with statistical analysis software (SPSS software platform) to determine whether the criteria are met for each measurement (i.e., SUS ≥ 70; UES ≥ 70; CVI > 0.80) [38]. The criteria will be analyzed by computing the average of the rating scores proposed by participants for each Likert item and finding the degree of inter-rater agreement on the IDDEAS system attributes (i.e., prompt/alert provided in system user-interface).

The sensitivity, specificity, and relevance of the IDDEAS system for ADHD diagnosis and treatment will also be assessed based on overall percentage of agreement among participants on appropriate diagnosis, as well as the proposed biopsychosocial treatment plan. A mixed model logistic regression will be used with correct diagnosis as the dependent variable, decision support (yes or no) and patient status (ADHD or non-ADHD) as fixed effects.

#### IDDEAS CDSS system modification and refinement

Between the two phases of the IDDEAS evaluation study, adjustments to the measurement tools and the system will be made. Based on the results of the vignette-based evaluation, prior to the live patient evaluation, adjustments to the questionnaires, the CDSS content provided for practitioners, and the overall design of the user-interface will be adjusted as necessary.

#### Outcomes

The primary outcome of the study will be the clinical utility of the IDDEAS CDSS for diagnosis and treatment of child and adolescent mental health disorders. The primary outcome will be measured by reviewing participants’ clinical diagnosis and treatment plans as a measure of sensitivity and specificity when using the CDSS compared to when not using the CDSS, upon completion of both phases of the evaluation.

The secondary outcomes of the study will be subjective measures. The three secondary outcome measures are perceived clinical usability, perceived clinical relevance and validity, as well as perceived appropriateness of the IDDEAS CDSS. The perceived clinical usability of the CDSS will be measured using the system usability scale (SUS) [33, 39, 40]. The perceived appropriateness of the CDSS will be measured using the user-engagement scale (UES) [41–43]. The perceived clinical relevance and validity of the system’s user-interface will be measured using the content validity index (CVI) [44].

All outcomes will be measured directly following both phases of the evaluation of the IDDEAS CDSS (i.e., within 24 h).

### Stage 4: Implementation & Dissemination

From the outset of the IDDEAS project, a scientific communication and dissemination plan will be implemented in line with both the Golden Road and the Green Road for dissemination. Findings and relevant study information will be regularly disseminated to the academic community, healthcare professionals, service-user organizations and the general public at conferences, congresses, workshops, and through social-media platforms (i.e., Twitter, Facebook, Instagram, etc.). Scientific communication will be disseminated as peer-reviewed publications in both national and international journals annually. Practical information on the IDDEAS CDSS will also be made available for all end-users, including an informative website, online tutorial and user guides. Prior to implementation of IDDEAS, preselected Consortium members and clinical experts will guide trial participants through training courses in order to qualify the clinicians as trainers for future IDDEAS End-User training courses. Follow-Up reviews and support meetings will be held to receive the clinicians’ feedback on using the IDDEAS CDSS. IDDEAS CDSS workshops will be held at the Norwegian CAMHS annual congress (i.e., N-BUP Kongressen).

## Discussion

IDDEAS will utilize qualitative and quantitative methods to determine whether the implementation of a clinical guideline and data-driven CDSS model in CAMHS will improve the quality of diagnoses and treatment of child and adolescent mental health disorders. The inclusion of two phases of evaluation within the IDDEAS trial will allow for a thorough assessment of the specific aspects of the CDSS that are suitable and those that need to be addressed for improvement of clinical care based on clinician’s subjective perception, as well as objective statistical analysis.

IDDEAS’ expected impacts include, but are not limited to, improved use of available health data, integration of predictive interventions in care, better management of complex clinical situations in child and adolescent mental health, enhanced collaboration among stakeholders involved in patient care, and amplified inter-service coordination in management of patient’s health. Furthermore, IDDEAS will help to improve patients’ understanding of the clinical decision- making involved in their treatment, as well as help ensure greater participation and improved transparency for the patients’ families. Overall IDDEAS will improve the quality of mental health care for children and adolescents by using innovative data-analytics within the CDSS model to provide support to clinicians that is evidence-based and customized to meet the needs of each individual patient. With quality improvement of clinical standards and enhanced precision of care, IDDEAS will also improve the efficiency of practices, allowing for more patients to be seen and receive a diagnosis in a timely-manner.

Our research will provide a comprehensive understanding of how to approach the use of a CDSS as a novel innovation for CAMHS. All limitations and challenges faced through the processes of designing, modelling, evaluating and testing the implemented IDDEAS CDSS model, can serve as valuable learning opportunities for future CDSS implementations in CAMHS.

## Data Availability

The datasets used and/or analyzed during the current study are available from the corresponding author on reasonable request.

## Abbreviations

ADHD: Attention-deficit/hyperactivity disorder
ASD: Autism spectrum disorder
BUP: Barne-og ungdompsykiatrisk poliklinikk/child and adolescent psychiatric clinic
CAMHS: Child and adolescent mental health services
CCQ: Clinical competence question
CDSS: Clinical decision support system
CDS: Clinical decision support
CVI: Content validity index
DBD: Disruptive behavioural disorders
DPIA: Data protection impact assessment
EHR: Electronic health record
ICT: Information and communication technologies
IDDEAS: Individualized digital decision assist system
NFR: Norsk forskningsrådet/Norwegian research council
OWL: Web ontology language
PCP: Primary care provider
PID: Personal identifiers
RCT: Randomized controlled trial
SUS: System usability scale
UES: User-engagement scale
WHO: World health organization
YLD: Years lived with disability
